The article "Placental serotonin: implications for the developmental effects of SSRIs and maternal depression" was published in 2013. Journal: Front Cell Neurosci.

# Placental serotonin: implications for the developmental effects of SSRIs and maternal depression

**DOI:** 10.3389/fncel.2013.00047

**Published:** 2013-04-23

**Authors:** Juan C. Velasquez, Nick Goeden, Alexandre Bonnin

**Affiliations:** Department of Cell and Neurobiology, Keck School of Medicine, Zilkha Neurogenetic Institute, University of Southern CaliforniaLos Angeles, CA, USA

**Keywords:** placenta, serotonin, SSRI, tryptophan, depression, fetal programming, fetal brain, serotonin transporter

## Abstract

In addition to its role in the pathophysiology of numerous psychiatric disorders, increasing evidence points to serotonin (5-HT) as a crucial molecule for the modulation of neurodevelopmental processes. Recent evidence indicates that the placenta is involved in the synthesis of 5-HT from maternally derived tryptophan (TRP). This gives rise to the possibility that genetic and environmental perturbations directly affecting placental TRP metabolism may lead to abnormal brain circuit wiring in the developing embryo, and therefore contribute to the developmental origin of psychiatric disorders. In this review, we discuss how perturbations of the placental TRP metabolic pathway may lead to abnormal brain development and function throughout life. Of particular interest is prenatal exposure to maternal depression and antidepressants, both known to alter fetal development. We review existing evidence on how antidepressants can alter placental physiology in its key function of maintaining fetal homeostasis and have long-term effects on fetal forebrain development.

## Introduction

There is a wealth of evidence suggesting that serotonin (5-HT) plays a critical role in many neurodevelopmental processes. Basic and epidemiological studies link disruption of the 5-HT pathway to a host of developmental and functional disorders, yet direct evidence of the molecular mechanisms underlying these perturbations remains lacking, especially in humans. Studies in animal models have indicated that 5-HT is a key modulator of neuronal cell proliferation, migration, and brain wiring during fetal and early postnatal development (Brezun and Daszuta, 1999, 2000, 2008; Azmitia, 2001; Kindt et al., 2002; Banasr et al., 2004; Bonnin et al., 2007). Furthermore, genetic and environmental disruption of 5-HT receptor function during critical periods of fetal brain development in mice lead to behavioral abnormalities throughout life, such as adult anxiety disorders (Gaspar et al., 2003; Holmes et al., 2003a,b; Ansorge et al., 2004; Nordquist and Oreland, 2010; Morelli et al., 2011; Garbett et al., 2012; Malkova et al., 2012). Interestingly however, there is sparse evidence of specific associations between 5-HT receptor gene mutation or dysfunction and mental illness in humans (Gingrich and Hen, 2001; Gaspar et al., 2003; Segman et al., 2003).

The article "Placental serotonin: implications for the developmental effects of SSRIs and maternal depression" was published in 2013. Journal: Front Cell Neurosci.

Generally weak phenotypes in single receptor knockout mice and the existence of 15 different receptor subtypes for 5-HT suggest that genetic alteration of one specific subtype may be compensated for by the presence of other pharmacologically and functionally similar receptors (e.g., 5-HT1B and 5-HT1D receptors; see Van Kleef et al., 2012). Basic studies were able to alter function of several receptors simultaneously during restricted, critical time periods, thus potentially preventing compensatory signaling through other receptors and leading to clear phenotypes (Ansorge et al., 2004; Bonnin et al., 2007).

What is common to all receptor subtypes is their endogenous ligand, 5-HT. Therefore, altered 5-HT tissue concentration may lead to generalized disruption of signaling through more than one receptor type simultaneously. This possibility is supported by dramatic effects from the pharmacological disruption of 5-HT synthesis in early experiments, contrasting with mild effects of single receptor knockout models (Van Kleef et al., 2012).

Recent results show that 5-HT signaling, and thus extracellular levels of 5-HT, play a crucial role in the thalamocortical wiring of the fetal forebrain by affecting netrin-1 mediated axonal guidance (Bonnin et al., 2007, 2011). Thus, altered 5-HT concentration in the fetal brain tissue, in addition to signal/receptor interaction, may have far-reaching developmental and functional consequences (Bonnin and Levitt, 2012). A recent study showed that the fetal forebrain accumulates placentally derived serotonin during early pregnancy (Bonnin et al., 2011), a period during which axons are experiencing active outgrowth and guidance. The role of placental metabolism of 5-HT from maternally derived TRP, its potential genetic and environmental perturbations, and their downstream consequences are currently under intense investigation.

## 5-HT and fetal brain development

Serotonergic neurons are one of the most ubiquitous circuits in the mammalian brain, forming early during fetal development, and innervating essentially the entire central nervous system. The early presence of 5-HT, as well as the proposed maternal origin of 5-HT, has led to the hypothesis that 5-HT may be an essential growth and regulatory factor for the fetal brain during critical periods of development (Lauder and Krebs, 1976; Lidov and Molliver, 1982; Gaspar et al., 2003; Bayard et al., 2007; Bonnin et al., 2011; Migliarini et al., 2012). This is supported by the idea that disruption of the 5-HT signaling system is a key developmental component for a number of neuropsychiatric disorders, such as schizophrenia, affective disorders, anxiety, and autism (Chugani et al., 1999; Whitaker-Azmitia, 2001; Sodhi and Sanders-Bush, 2004; Bonnin and Levitt, 2012). Genetic mouse models have shown that excess levels of 5-HT in the brain, obtained by knocking out the transporter (SERT; *Slc6a4*) or monoamine oxidase-A *(MAO-A)* genes, which are involved in the re-uptake and degradation of 5-HT, respectively, lead to abnormal development of topographically organized whisker-barrel fields in the somatosensory cortex (Cases et al., 1996; Persico et al., 2001). Furthermore, recent studies have shown that increased activity of the serotonergic pathway may lead to abnormal cortical development and neuronal migration (Janusonis et al., 2004; Riccio et al., 2009). On the other hand, 5-HT depletion through the use of *Pet1* knockout mice, in which there is a dramatic reduction of serotonergic neuron number and differentiation, shows no identifiable gross brain malformations, despite evidence of later behavioral and functional deficits (Hendricks et al., 2003; Liu et al., 2010). Similarly, targeted inactivation of *tryptophan hydroxylase 2 (Tph2)*, the rate-limiting enzyme for the synthesis of 5-HT specifically in the brain, in the mouse model has been demonstrated to produce behavioral and functional deficits. However, lack of 5-HT did not lead to obvious cellular or histological abnormalities in the brain (Savelieva et al., 2008; Alenina et al., 2009; Yadav et al., 2009). Nevertheless, the more recent analysis of a knock-in mouse line, in which the brain-specific *Tph2* gene was replaced by an eGFP reporter, showed significant abnormalities in serotonergic innervation in several regions of the rostral brain (Migliarini et al., 2012). Combined, these data suggest that specific circuits are finely tuned to 5-HT during their initial formation, including the serotonergic system itself. The next logical question is to determine if, and how, 5-HT signaling during development is impacted by genetic and environmental perturbations shown to be associated with increased risk of neuropsychiatric disorders.

The article "Placental serotonin: implications for the developmental effects of SSRIs and maternal depression" was published in 2013. Journal: Front Cell Neurosci.

Recent work suggests that the maternal and placental source of 5-HT may be a critical link between early genetic and environmental perturbations and their impact on fetal brain development. Consequently, exposure to pharmacological or environmental insults, combined with genetic factors that disrupt maternal or placentally derived 5-HT may have profound and long-lasting consequences on the developing brain, leading to a host of neuropsychiatric disorders thought to have developmental origins.

In the next section, we discuss how particular environmental and pharmacological insults such as exposure to maternal depression and antidepressants during pregnancy may impact fetal brain development, taking into account the potential effects on the maternal-fetal interface function.

## Prenatal exposure to maternal depression and antidepressants, effects on fetal brain development and long-term consequences

Major Depression Disorder (MDD) is a devastating mood disorder that indiscriminately affects individuals of all backgrounds and ages, and is common even in women during gestation. In fact, the prevalence of MDD is about 15% during pregnancy, and Selective Serotonin Reuptake Inhibitors (SSRIs) are the primary pharmacologic intervention (Oberlander et al., 2006). Despite an unclear safety profile and a lack of well-controlled safety studies, an estimated 13% of pregnant women are prescribed an SSRI antidepressant during all or part of their pregnancy (Cooper et al., 2007). This common off-label use is warranted for its beneficial effects of improving maternal mood and relieving symptoms of depression, which presumably lead to better pregnancy outcomes. Due to their high use and unknown safety, there is high surveillance of SSRIs by the US Food and Drug Administration, which has placed some SSRIs in Pregnancy Category D, indicating demonstrated risks to the fetus (Greene, 2007).

Recent epidemiological studies suggest that fetal exposure to maternal SSRI therapy is implicated in disturbing several physiological and cognitive domains during fetal development. Their prescribed use is associated with increased prevalence of preterm delivery, intrauterine growth restriction, and neurobehavioral disturbances in infants (Oberlander et al., 2009). Additionally, fetal SSRI exposure has been shown to increase risks of Postnatal Adaptation Syndrome, low Apgar scores, Persistent Pulmonary Hypertension of the Newborn, long-term changes in cardiac morphology and physiology, gastrointestinal abnormalities, Autism Spectrum Disorders, and postnatal language learning deficits in humans (Figure 1). (Cohen et al., 2000; Simon, 2002; Laine et al., 2003; Källén, 2004; Chambers et al., 2006; Levinson-Castiel et al., 2006; Oberlander et al., 2006; Cooper et al., 2007; Louik et al., 2007; Talge et al., 2007; Calderon-Margalit et al., 2009; Lund et al., 2009; Merlob et al., 2009; Pedersen et al., 2009, 2010; Hadjikhani, 2010; Kornum et al., 2010; Reis and Källén, 2010; Croen et al., 2011; Haskell et al., 2012; Jimenez-Solem et al., 2012; Nijenhuis et al., 2012a,b; Nordeng et al., 2012; Weikum et al., 2012; Yonkers et al., 2012).

**Figure 1:** **(A)** Treatment of maternal depression with SSRIs is associated with varying pregnancy outcomes. While every gestational stage of SSRI exposure has been implicated in increased risks for cognitive, physiological, or developmental teratogenicity, the period of exposure is an important factor that appears to influence clinical outcomes in the offspring. We limited this list to outcomes that have been the focus of several epidemiological studies in recent years and for which differential exposure data during pregnancy was available. **(B)** Untreated maternal depression and stress have been associated with several risks that affect cognitive and developmental outcomes. While associations are not generally correlated to specific trimesters, exposure to untreated maternal depression or stress during pregnancy pose adverse risks to fetal health and development. *Study Selection and Data Extraction* Studies were selected if they had clearly identified maternal SSRI exposure for specific trimesters of pregnancy and assessed neonatal outcomes. Epidemiological studies that included medium-to-large number samples exposed to different SSRI drugs were selected. Direct comparison of absolute odds ratio values across these studies is not possible due to varying specific study designs, adjustments for level of maternal depression and various sociodemographic and lifestyle factors, drug dosages, length of exposure, and SSRI treatment options. ^*^PPHN, Persistent pulmonary hypertension of the newborn.

The article "Placental serotonin: implications for the developmental effects of SSRIs and maternal depression" was published in 2013. Journal: Front Cell Neurosci.

Leaving maternal MDD untreated to avoid the potential teratogenicity of SSRIs also poses significant risks. The anguish and psychological distress accompanied by untreated MDD induces considerable maternal stress, one of the earliest adverse experiences with long-term effects on the offspring. Several animal and human studies show that maternal stress or depression disrupt fetal neurobehavioral development and affect cognitive, emotional and behavioral outcomes throughout childhood (Peters, 1990; Hayashi et al., 1998; Talge et al., 2007; Homberg et al., 2010). Children exposed to the stress induced by depressed mothers are also at increased risk of developmental delay, impaired language development, and even low IQ scores (Figure 1) (Deave et al., 2008; Paulson et al., 2009). The impact of maternal depression on newborns has effects that last beyond infancy, as one-third of school-aged children of depressed mothers suffer from depression and anxiety disorders (Pilowsky et al., 2006). Beyond childhood, animal studies have shown that neonatal SSRI exposure suppresses adult serotonergic signaling and elicits depressive- and anxiety-like behaviors in adulthood (Ansorge et al., 2008; Shanahan et al., 2009).

The article "Placental serotonin: implications for the developmental effects of SSRIs and maternal depression" was published in 2013. Journal: Front Cell Neurosci.

Maternal depressive states and prenatal exposure to SSRIs both alter fetal health. For the developing fetus, associated risks stem from both the untreated illness and the treatment itself, underscoring a therapeutic risk-benefit dilemma: SSRI treatments that safeguard maternal health have adverse effects on the developing fetus, but leaving maternal depression untreated also poses various significant, adverse risks.

Several perspectives have been offered to account for how some psychiatric disorders may arise from the disruption of particular neurotransmitter systems during development. Disruption during sensitive developmental periods may have lasting effects expressed during adulthood, and since 5-HT signaling participates in several developmental programs (see above), dysfunction of the 5-HT system may be implicated in the etiology of several mental disorders in humans, particularly in MDD. Genetic studies in mice show that transient developmental disruption the 5-HT system by exposure to SSRIs results in long-term behavioral abnormalities and increased anxiety in adult offspring (Ansorge et al., 2004, 2008; Maciag et al., 2006; Oberlander et al., 2008). Not only does neonatal SSRI exposure reduce serotonergic signaling, but also elicits a down regulation in midbrain expression of *Tph2*, an essential enzyme in the serotonin synthesis pathway (see above, Maciag et al., 2006).

As mentioned above, studies in animal models point to evidence that 5-HT influences mammalian nervous system development. Disruption of 5-HT signaling has several important implications, namely in the modulation of axonal guidance mechanisms that establish precise fetal brain circuits (Gross et al., 2002; Bonnin et al., 2006, 2007). Because embryonic thalamocortical axons (TCAs) accumulate 5-HT and express a range of 5-HT receptors as well as SERT, serotonin is able to shape the outgrowth and synaptic connectivity of their projections (Bonnin et al., 2012). SSRIs target and block SERT with high affinity, and have been shown to directly affect serotonergic modulation of TCA responses to the guidance cue netrin-1 *in vitro.* The presence of the SSRI citalopram (R/S enantiomers mixture) switched TCA response to netrin-1 from attraction to repulsion, impacting the direction of their projections (Bonnin et al., 2012). Moreover, mice with genetically disrupted SERT function, which may serve as a model for chronic SSRI exposure, display changes in neuronal cytoarchitecture, 5-HT function and neurobehaviors, all components that have developmental origins (Oberlander et al., 2009). In addition, genetic studies in mice show that disruption of 5-HT receptors expression during a restricted period of pre- and postnatal development results in long-term behavioral abnormalities (Gross et al., 2002). Taken together, these results suggest that SSRIs could induce topographical shifts in important circuits of the fetal brain, thus constituting a possible mechanism that gives rise to certain mental illnesses by altering circuit-formation and ultimately, proper brain function later in life.

The article "Placental serotonin: implications for the developmental effects of SSRIs and maternal depression" was published in 2013. Journal: Front Cell Neurosci.

## Impact of SSRIs on fetal development may depend on routes of exposure during pregnancy

The placenta is essential for ensuring the growth and survival of the fetus during development. Not only does it support fetal homeostatic functions, but also serves as the essential source of 5-HT for the fetal forebrain during a transient, critical period of development (Bonnin et al., 2011; Bonnin and Levitt, 2012). The placenta is able to synthesize 5-HT from a maternal TRP precursor in both mice and humans (Bonnin et al., 2011; Bonnin and Levitt, 2012; Goeden and Bonnin, 2013). This exogenous source of 5-HT is available to the fetal brain during developmental milestones including cortical neurogenesis, cell migration, and circuit formation (Bonnin et al., 2011). Therefore, proper placental function during gestation may be essential for the 5-HT modulation of neurodevelopment.

The placenta may play a major role between SSRIs exposure and their associated teratogenicity during gestation. Since the fetal brain acquires placenta-derived 5-HT during a critical period of widespread axonal outgrowth, the effects of SSRIs on fetal brain development may be through an indirect pathway that affects proper placental physiology, resulting in indirect, downstream effects on the fetus. Although it is not clear whether SSRI exposure induces physiological changes in the placenta, its high expression of SERT support the notion that SSRIs would retain their high binding affinity in this organ (Ganapathy et al., 1993; Yavarone et al., 1993; Shearman et al., 1998; Verhaagh et al., 2001). If blocking SERT function alters placental 5-HT synthesis and/or transport to the fetus, or maternal 5-HT degradation, SSRI treatments could be teratogenic primarily by altering placental physiology. The placenta's key function of maintaining fetal homeostasis may thus be compromised and have long-term effects on fetal forebrain development.

Alternatively, SSRIs may be able to readily cross the placenta and enter the fetal circulation, where they could directly target the developing brain's serotonergic system. While there is some evidence of SSRIs crossing the placenta, studies have focused on umbilical cord concentrations at birth in humans (Hostetter et al., 2000; Hendrick, 2003; Sit et al., 2011). Several commonly used SSRIs such as Citalopram, Fluoxetine, and Paroxetine were shown to cross the placental barrier at term, with various efficiencies (e.g., mean ratios of umbilical cord to maternal serum concentrations ranged from 0.29 to 0.89) (Hendrick, 2003). These studies give a snapshot of maternal-fetal SSRI transplacental transport at birth; however, there is no data earlier in gestation, particularly when the fetal brain may be most susceptible to disruptions of 5-HT signaling. Such data is difficult to obtain in humans, rendering studies in animal models as crucial and necessary to providing key insights.

The article "Placental serotonin: implications for the developmental effects of SSRIs and maternal depression" was published in 2013. Journal: Front Cell Neurosci.

The impact of SSRIs on fetal brain development may therefore result from direct actions on the fetal brain, indirect actions on placental or maternal physiology or, more likely, a combination of all these routes (Figure 2). Ongoing efforts to measure transplacental transfer and effects on placental physiology of SSRIs throughout the course of pregnancy in mice, and to determine the drugs biodistribution in the fetus, will help determining precisely how they affect fetal brain development.

**Figure 2:** **The effects of SSRIs on fetal brain development may be through direct (A) or indirect pathways that affect placental (B), maternal (C), or both maternal and placental physiology (D), ultimately resulting in downstream effects on the fetus.** Direct effects **(A)** suggest that SSRIs readily cross the placenta and enter the fetal circulation, where they would directly target the developing brain's serotonergic system. Alternatively, physiological changes in the placenta **(B)**, or delivery of maternal factors essential for the developing fetal brain **(C)** may be affected through indirect pathways. The combination of both direct and indirect pathways inducing adverse effects on the fetal brain may also be possible **(D)**. Under the influence of varying s maternal, fetal and placental (maternal-fetal combination) genetic susceptibilities (DNA double helix), the effects of SSRI exposure at different pregnancy stages may lead to diverse developmental outcomes.

## A concluding perspective on the role of 5-HT on the neurodevelopmental programming of mental diseases

Transient disruption of essential signaling events during critical developmental periods may have lasting effects that are expressed throughout life. The serotonergic system steers neurodevelopment through the key modulation of neurogenesis, cell migration, and brain wiring that give rise to proper brain function. With a diversity of molecular targets on which to focus, it makes sense that perturbations of 5-HT signaling have been implicated in the pathogenesis of diverse neurodevelopmental disorders. The perturbations of the 5-HT neurotransmitter system during development, whether directly on the fetal brain or on its placental modulation during early gestation, may have long-lasting developmental and physiological consequences. Risk factors, both genetic and environmental, that alter 5-HT concentration in the fetal brain tissue may thus ultimately pose far-reaching functional consequences throughout life.

The article "Placental serotonin: implications for the developmental effects of SSRIs and maternal depression" was published in 2013. Journal: Front Cell Neurosci.

Fetal exposures to SSRIs and maternal stress induced by MDD are early exposures that have been associated with various diseases affecting physiological and cognitive domains. The heterogeneity and diversity of different disease outcomes is informed by the length and developmental period of adverse exposures, in addition to fetal genetic susceptibilities. Together with the altered fetal brain 5-HT signaling caused by SSRI exposure in different stages, the influence of maternal, fetal and placental (maternal-fetal; see Figure 2) genetics could possibly lead to different disease states. The manifestation of several mental disorders associated with serotonin dysfunction, namely MDD, ASD, and other psychiatric illnesses may thus require multiple events of environmental, genetic, and their interactions, to occur.

While the associated risks from fetal SSRI exposure continue to be elucidated, the mechanisms of 5-HT neurodevelopmental disruptions, and how they ultimately lead to adult-onset disorders need further study. There is also a clinical demand for effective and safe treatment of maternal MDD, taking into consideration the effects of drug therapy on the safety of the developing fetus.

### Conflict of interest statement

The authors declare that the research was conducted in the absence of any commercial or financial relationships that could be construed as a potential conflict of interest.
